# Effects of Outlets on Cracking Risk and Integral Stability of Super-High Arch Dams

**DOI:** 10.1155/2014/312827

**Published:** 2014-07-23

**Authors:** Peng Lin, Hongyuan Liu, Qingbin Li, Hang Hu

**Affiliations:** ^1^State Key Laboratory of Hydroscience and Engineering, Tsinghua University, Beijing 100084, China; ^2^School of Engineering, The University of Tasmania, Hobart, Australia

## Abstract

In this paper, case study on outlet cracking is first conducted for the Goupitan and Xiaowan arch dams. A nonlinear FEM method is then implemented to study effects of the outlets on integral stability of the Xiluodu arch dam under two loading conditions, i.e., normal loading and overloading conditions. On the basis of the case study and the numerical modelling, the outlet cracking mechanism, risk, and corresponding reinforcement measures are discussed. Furthermore, the numerical simulation reveals that (1) under the normal loading conditions, the optimal distribution of the outlets will contribute to the tensile stress release in the local zone of the dam stream surface and decrease the outlet cracking risk during the operation period. (2) Under the overloading conditions, the cracks initiate around the outlets, then propagate along the horizontal direction, and finally coalesce with those in adjacent outlets, where the yield zone of the dam has a shape of butterfly. Throughout this study, a dam outlet cracking risk control and reinforcement principle is proposed to optimize the outlet design, select the appropriate concrete material, strengthen the temperature control during construction period, design reasonable impounding scheme, and repair the cracks according to their classification.

## 1. Introduction

Arch dam has been constructed for water storage reservoir since early times such as the Kurit dam constructed in Iran in the 13th century, the Elche dam in Spain in the 17th century, and the Pontalto dam in Italy in the 17th century [1, 2]. Since the middle of the 19th century, the number of arch dams has greatly increased [1]. Nowadays, the arch dam has attracted extensive researches in structural engineering health monitoring [3–5], intelligent cracking control [6–8], and computer simulation [9]. Design and optimization of the arch dam and health monitoring of the dam structural performance and behaviour under extreme loadings are just being unfolded throughout these researches. China is abundant in hydraulic resource, which is estimated to be 680 million kilowatt theoretically and 370 million kilowatt available to be exploited. Both of them rank the first in the world. For sustainable development of clean energy, a series of super-high arch dams have been constructed in southwestern China including the Xiaowan, Xiluodu, Jinping I, and Laxiwa arch dams with heights of 294.5 m, 285.5 m, 305 m, and 251 m, respectively [10, 11]. Nowadays, the techniques for constructing the general arch dam with a height less than 200 m may become mature but the construction of the super-high arch dam with a height of around 300 m, such as the Xiaowan, Xiluodu, and Jinping I dams, still faces many challenges, for example, the cracking risk and integral stability of the dam body and the reinforcement measure and mechanical behaviour of the complex dam foundations consisting of jointed or altered rock mass and atypical faults. During the construction and service of the arch dams, cracks may develop in the dam body due to internal and external temperature variation, concrete shrinkage, differential abutment foundation deformation, previous earthquake, or other reasons [11–16]. Although these cracks may only propagate to a limited depth in the dam body, they may weaken the overall loading capacity of the arch dams.

Moreover, the super-high arch dams tend to layout more ancillary structures such as outlets for various purposes, for example, flood discharging, sediment removal, silt scouring, and reservoir emptying, which are usually distributed in a relatively high density in the dam body, as shown in Figure 1. During the service of the super-high arch dams, stresses may concentrate around the outlets causing cracking of the dam body [15, 16], which poses further potential threats to the integral stability of the arch dams. In the past, designers mainly focused on the dam body [17, 18] but paid less attention to the effects of the outlets on the integral stability of the dams [19–25]. Although there are studies proving that cracks around outlets have little effect on the integral stress status and loading condition of the dam [11, 15, 23, 25], in the long-term conditions, the pore water pressure may stimulate the cracks around the outlets to propagate and coalesce with those caused by other factors mentioned above, which may result in greater risk to the integral stability of the super-high arch dam.

Three kinds of theoretical analysis are adopted in literatures to analyze effects of outlet cracking on the integral stability of the super-high arch dams. (1) Plane stress analysis: if the outlet opening is relatively small compared with the whole dam body and the minimum distance between the centre of the outlet and the dam foundation is not less than three times of the width of the outlet, only local stress distributions of the dam will be affected by the outlet. Thus, appropriate two-dimensional (2D) section of the outlet may be selected for plane stress analysis. (2) Linear elastic analysis: in the area where tensile stress exceeds the strength of concrete, it is assumed that the concrete completely cracks and reinforcement bar bears all the tensile stress. Linear elastic analysis is usually suggested for the preliminary design of the concrete dam and its components and usually leads to a large safety factor in design [17, 18], which cannot often guarantee construction quality and economic benefit. (3) Nonlinear analysis: when induced tensile stress reaches the tensile capacity of concrete, cracks appear in the dam concrete, which causes part of the excess stress to be released and the others are gradually shifted to the reinforcement bar. In this case, the stress near the crack tip remains below the tensile capacity of concrete. As the load increases, the existing crack may further open and propagate. At the same time, secondary and tertiary cracks may appear due to the bonding effect between the reinforcement bars and the concrete when stress in adjacent area reaches the tensile capacity of concrete [26–32]. Three-dimensional (3D) numerical simulation is probably the most popular nonlinear analysis method, which has now been applied widely to analyze the integrity and stability of the high arch dams [11, 12, 22, 25] and the associated underground water transmission tunnels [28]. (4) The Saint-Venant principle: submodel method can be adopted to analyze the dam outlets according to the Saint-Venant principle, that is, when the actual load is replaced by an equivalent load, stress, and strain only changes in the loading area. The specific steps are as follows: (a) analyze the integral model of the super-high arch dam using finite element method with coarser mesh; (b) cut out a submodel with the outlets from the integral model to establish a submodel with finer mesh; (c) calculate the displacements of all points on the boundary of the submodel by interpolating the results from the step (a) and use the calculated displacements as the initial boundary conditions of the submodel for the analysis in the next step; and (d) analyze the submodel using the finite element method analysis according to the boundary conditions calculated from the step (c).

However, most of the analyses available in literatures are conducted for the dams without sufficient considerations of outlets, which lead to a large gap between the obtained and actual stresses and/or displacements for the dams and may adversely affect the dam design, construction, and optimization processes. In sum, the effect of the outlets on working condition of the super-high arch dam is still a blank area worthy of further studies.

In this study, the status, reason, and consequence of the outlet cracking in the Goupitan and Xiaowan super-high arch dams are first discussed. The effects of the outlets on the deformation, stress, cracking risk, and overall stability of the Xiluodu super-high dam are then analyzed using a finite element method. Finally, a dam outlet cracking risk control method is proposed on the basis of the outlet cracking mechanism identified above to ensure the safety and stability of the super-high arch dams.

## 2. Case Studies on Dam Outlet Cracking

### 2.1. Outlet Cracking at the Goupitan Arch Dam

#### 2.1.1. Introduction to the Outlets in the Goupitan Arch Dam

The Goupitan high arch dam (Figure 1) is constructed on the Wujiang River in Guizhou Province, southwestern China. The dam is a double curvature concrete arch with a maximum height of 230.5 m, a ratio between thickness and height of 0.216, and a crest length of 552.55 m. There are 6 flood discharging upper outlets, 7 flood discharging middle outlets, 2 reservoir empting bottom outlets, and 4 temporary diversion bottom outlets, as shown in Figure 1. The elevation level (EL) of the upper outlets is 617 m above the sea level and the size of each outlet is 12 m × 13 m (width × height). The size of the middle outlets is 7 m × 6 m. The numbers 1, 3, 5, and 7 middle outlets have plat bottom, and their entrances are at EL 550 m. The numbers 2 and 6 middle outlets hold an exit jet angle of 25 degree and its entrance is at EL 543 m. The number 4 middle outlet holds an exit jet angle of 10 degree and its entrance is at EL 546 m. The size of the control section in the reservoir empting bottom outlets is 3.8 m × 6 m and that in the temporary diversion bottom outlets is 6.5 m × 8 m. The entrance of the bottom outlets are at EL 490 m. The upper surface of the outlets is built with C35 abrasion-resistant concrete, which extends from the surface to 1-metre-deep inside. The reservoir empting bottom outlets and diversion bottom outlets are built with C50 abrasion-resistant concrete, and the transition zone of C50 and C18035 is built with the C35 concrete. C18035 is also used for the construction of the temporary diversion bottom outlets, the reservoir empting bottom outlets, and the flood releasing middle outlets of nonspillways in the numbers 11 to 17 dam monoliths.

#### 2.1.2. Outlet Cracking Status

Three groups of defects were discovered in the Goupitan concrete arch dam at the end of May 2008. The first one was the peripheral fractures observed near the number 1 reservoir empting bottom outlets, as shown in Figure 2. The second one was the cracks near the foundation corridor in the number 19 dam monolith. The last was the cracks near the lift platform of the number 2 reservoir empting bottom outlets in the number 14 dam monolith, as shown in Figure 3. Among them, the peripheral fractures near the bottom outlets (Figures 2 and 3) have the largest scale and most harm the integral stability of the dam. Correspondingly, these cracks are classified, which are summarized into Table 1 together with their characteristics and subsequently adopted reinforcement measures.

Furthermore, the status of the peripheral fractures near the reservoir emptying bottom outlets is highlighted here. The first series of cracks appeared at the end of November 2006 in the surfaces of the number 13 dam monolith at EL 491 m for the number 1 reservoir emptying bottom outlet and the number 14 dam monolith at EL 497 m for the number 2 bottom outlet, as shown in Figure 2 and Table 2. Crack-limiting reinforced nets and chemical grouting pipe-system are installed to control and repair these cracks. Besides them, the other reinforcement method for the cracks mentioned hereafter includes filling in cracks using preshrinkage mortar, drilling stress release hole, and installing double-layer crack-limiting steel bar. After the construction of the bottom outlets but before the grouting of the transverse joint in the number 9 grouting zone (from EL 479.0 m to EL 488.0 m), all the bottom outlets are examined and new second series of cracks are found in the side walls and floors, as shown in Figures 2 and 3(a) and Table 1. Then visual inspection and water pressure test of transverse joints are carried on all the bottom outlets and the sonic wave test is adopted for deep investigation. The third series of cracks are identified, as summarized in Table 1.

Moreover, there are local cracks in the numbers 1, 2, and 4 diversion bottom outlets which coalesce with the transverse joints at a distance of about 10 m from the upstream surface. These cracks are rather long but the width is about 0.2 mm. The depth of the cracks in the floor and roof of the bottom outlets is shallow, and the majorities of them are less than 1 m. However, the cracks in the side wall are somehow deeper and the greatest depth is larger than 2.8 m.

In sum, the number of cracks in the different outlets ranges from 13 to 21 and the majority of them is longitudinal (Figure 2(c)) according to the results from the crack inspection.

#### 2.1.3. Reasons and Consequences of Outlet Cracking

Following the design requirements, the reservoir emptying and diversion bottom outlets are constructed with the C50 concrete so as to improve their abrasion-resistance capacity. As we know that the concrete has poor conductivity, high temperature gradients may be resulting in between the interior and the surface of the concrete structural elements or between parts of a concrete element during the sequential pouring phases. The temperature gradients may lead to tensile stresses, which may result in the young concrete cracking. In the Goupitan arch dam, the large amount of cements, the high temperature of hydration, and the hot weather in July during the construction of the bottom outlets lead to high temperatures inside the concrete. As the temperature of the concrete drops down sharply later, stress due to the temperature gradient of the concrete from inside to outside creates several cracks. As the time passes, the temperature of the concrete decreases continually and more and more cracks are appeared. In addition, if the conservation measures are not perfect; for example, the external concrete has not been supplied with sufficient water; the concrete surface will shrink generating further cracks. Actually, even if the upstream water level reaches EL 590.0 m, the resultant stresses at the reservoir discharging bottom outlets in the Goupitan arch dam are not more than the tensile or shear strengths of the C50 concrete. Thus, it is not necessary to use the C50 concrete during the construction of the abrasion-resistant layers of the bottom outlet from the point of view of the actual diversion capacity of the bottom outlets in the Goupitan arch dam.

In addition, the C35 concrete is used to construct the dams in the transition zone from the C50 to C18035 concretes. The shrinkage coefficients of the concretes differ from each other, which further contribute to the outlet cracking. The 3D finite element method was conducted by the design institute to analyze the stress and deformation of the Goupitan arch dam during the operation phases with and without outlet cracking. It is found that the integral stability of the dam is affected by the outlet cracking. The analysis results show that the existence of the cracks in the bottom outlets has little effects on the dam stress and displacement. During the operation phase, compressive and shear stress of crack is small, which indicates that the cracks will be closed and shearing slip will not occur. Even if water pressures and external loads are applied, the stress intensity factor at the tip of the cracks surrounding the outlets is still smaller than the fracture toughness *K*_IC_ of the concrete, illustrating that the crack will not continue to propagate.

### 2.2. Outlet Cracking at the Xiaowan Arch Dam

#### 2.2.1. Introduction to the Outlet in the Xiaowan Arch Dam

The Xiaowan arch dam (Figure 4) is constructed on the Meigong River in Nanjian County, Yunnan Province, southwestern China, which is a double curvature concrete arch dam with a maximum height of 294.5 m and a dam crest length of 905 m. The Xiaowan arch dam is the highest arch dam in operation in the world. As shown in Figure 4(a), three types of outlets, that is, the upper surface, middle diversion, and bottom exit outlets, are constructed in the Xiaowan arch dam to meet the needs of construction diversion, water impoundment, and generation of the first generation set. The cross section of the two bottom outlets is rectangular, each of them has a size of 6 m × 7 m, and their entrance ELs are 1020 m and 1050 m, respectively. The three middle diversion outlets are located in the numbers 21, 22, and 23 dam monoliths and numbered using the numbers 1, 2, and 3, respectively, from left to right in Figure 4(a). The maximum average diversion flow rate of single middle diversion outlet is designed as 1884 m^3^/s. The maximum average water flow speed is 45 m/s but it is 38 m/s at the centre of the middle diversion outlet. Taking the high speed and large amount of the diversion flow, the middle diversion outlets should be reinforced with fiber concrete. Below EL 1051 m, surfaces of the outlets are built with 0.6-metre-thick abrasion-resistant C2840W9010F90150 concrete.

#### 2.2.2. Outlet Cracking Status

The outlet cracking mainly occurs in the middle diversion outlets in the Xiaowan arch dam. Correspondingly, only the outlet cracking characteristics and reinforcement measures of the middle diversion outlets are summarized into Table 2. Since most of the cracks in the middle diversion outlets coalesce with the thermal cracks induced due to temperature gradient in the dam monoliths, these cracks are collected and classified according to the numbers of the dam monoliths in which the middle diversion outlets are located, as shown in detail in Table 2. Moreover, the distributions of outlet cracking in the number 22 dam monolith are depicted in Figure 4(b) while a snapshot of cracking near the number 2 middle diversion outlet is shown in Figure 4(c).

#### 2.2.3. Reasons and Consequences of Outlet Cracking

Because of the large displacement toward the upstream side of the arch dam when the water through the diversion outlets exceeds the designed amount, the large tensile stress near the upstream surface may be the main cause of the outlet cracking in the arch dam.

Cracks near the middle diversion outlets coalesce with those thermal cracks due to temperature gradient, which become the main source of water leakage. Our studies have shown that if the pore water pressure in the crack reaches 0.5 MPa, the crack may propagate. The bigger the aspect ratio, the smaller the pore water pressure needed for the crack to propagate. Currently the pore water pressure of 1.1 MPa in the cracks has led to a large amount of water leakage through the numbers 22 and 23 dam monoliths. If appropriate measures could not be taken timely to cut off the water source, the irregular cracks in the side wall of the outlets may propagate continually under the repeated pressing of the pore water in the cracks, which may harm the overall instability of the arch dam. The correspondingly crack reinforcement measures are listed in Table 2.

## 3. Effects of Outlets on Integral Stability of the Xiluodu Super-High Arch Dam

### 3.1. Introduction to the Xiluodu Super-High Arch Dam

In this section, effects of outlets on the working status of a 300 m high arch dam in the Xiluodu hydropower station are studied. The Xiluodu hydropower station is located on the Jinshajiang River, Leibo county, Sichuan Province, southwestern China. It is the second largest power station in the world and can produce 13.86 million kW of power, which is close to the capacity of the largest power station, that is, the Three Gorges hydroelectric power station. The principal structures consist of a double-curvature arch dam with a height of 285.5 m and a crest length of 603 m, spillway, underground powerhouse, and logway. The thickness of the dam is 14 m at crest and 60 m at the lowest foundation. There are 7 surface outlets, 8 deep outlets, and 10 diversion bottom outlets placed in the numbers 12~19 dam monoliths. The volume of the outlets counts for 2% of that of the whole dam.

The rock mass strata in the reservoir basin are clastic rock, carbonate rock, and basalt of Paleozoic, a small amount of metamorphic rock of Presinian and dolomite of Sinian [33, 34]. The depth of rock mass strongly unloaded due to the dam construction is generally less than 10 m. No strong weathered rock masses are founded in the reservoir generally except some thin weathering sandwiches located in some fault zones. Fresh rock and weak weathered rock mass is integral overall, which can mainly be classified as the type II rock mass. These rock masses have an acoustic velocity of 4800–5500 m/s, good uniformity, and weak permeability. Surface water drainage is unobstructed, groundwater level stays low, and natural slope has good stability. The foundation consists of several layers of fine basalts (e.g., P2*β*1 and P2*β*2) with an average thickness of about 25~40 m. The main weak zones are the interstrata bedding planes C9, C8, C7, C3, C2, and C1 and the intrastrata rupture belts Lc6 and Lc5 [24, 33]. These weak zones are filled with breccia, embedded sharp-angled fragments, coarse sand, and gravels, which are about 25 mm thick. The foundation of the dam is divided into a number of riverbed monoliths (e.g., from the numbers 14th to 19th monoliths), which are mainly composed of the type III1 rock masses with a few type III2 rock masses at the elevations 324.5 m and 328 m. The type III1 rock mass is either unweathered or a slightly weathered basalt. The physical-mechanical properties of the rock masses are listed in Table 5. The type III2 rock mass accounts for about 10~50% of the left and right steep slopes of the dam monoliths.

### 3.2. Numerical Model and Methodology

In this section, three-dimensional nonlinear finite element method is implemented to study the integral stability of the Xiluodu super-high arch dam with and without outlets under normal loading and overloading conditions. Some preliminary results from these analyses were reported previously in a conference paper ([35]) to exchange ideas with peers and collect feedbacks. However, this paper will focus on the nonlinear finite element analysis method and effects of the outlets on the deformation, stress, and integral stability of the Xiluodu super-high arch dam while the conference paper just briefly discussed the integral stability of the dam.

#### 3.2.1. Nonlinear Finite Element Analysis with Drucker-Prager Yield Criterion

The 3D finite element analysis adopts Drucker-Prager (D-P) yield criterion, which can be expressed in

(1) $$\begin{array}{c} f=\alpha I_{1}+J_{2}^{1/2}-H=0, \end{array}$$

where *I*_1_ is the first invariant stress, *J*_2_ is the second invariant stress, and *α* and *H* are material constants, which can be determined according to

(2) $$\begin{array}{c} \alpha =\frac{3tg\varphi }{\sqrt{9+12tg^{2}\varphi }},\;\;H=\frac{3c}{\sqrt{9+12tg^{2}\varphi }}, \end{array}$$

where *c* is cohesion and *φ* is friction angle. Equations (1) and (2) also show that the D-P criterion and the M-C (i.e., Mohr-Coulomb) criterion have the same expressions for the plane strain problem. In the *π* plane, the D-P circle has the intermediate values of circumstanced circle and inscribed circle of the M-C hexagon. Nonlinear elastoplastic finite element analysis can figure out conditions like plastic yield, subcritical fracture, and unstable extension and plot the unbalanced force and point safety factor contour in the upstream and downstream surface of the dam.

The stress adjustment process in the nonlinear finite element analysis with the D-P criterion can be listed as in the following: stress and strain of the initial point is set to be *σ*_0_ and *ε*_0_ and *f*(*σ*_0_) ≤ 0. For a given load step or iteration, the strain increment Δ*ε* of the point can be obtained by displacement method and correspondingly the stress can be calculated using

(3) $$\begin{array}{c} \sigma_{1}=\sigma_{ij}^{1}=D:\left(\varepsilon_{0}+\Delta \varepsilon \right), \end{array}$$

where **D** is the elasticity tensor. If *f*(*σ*_1_) > 0, then the stress needs adjustment. If plastic strain increment of the loading step or iteration is Δ*ε* ^*p*^, then the stress after adjusting can be written using

(4) $$\begin{array}{c} \sigma =\sigma_{ij}=D:\left(\varepsilon_{0}+\Delta \varepsilon -\Delta \varepsilon^{p}\right)=\sigma_{1}-D:\Delta \varepsilon^{p}. \end{array}$$

Transform the AC flow rule to incremental form approximately, which can be written into

(5) $$\begin{array}{c} \Delta \varepsilon^{p}=\Delta \lambda \frac{\partial f}{\partial \sigma }. \end{array}$$

Determine the representative value of ∂*f*/∂*σ* by *σ*_1_ using

(6) $$\begin{array}{c} f\left(\sigma \right)=0,\;\sigma =\sigma_{1}-\Delta \lambda D:{\frac{\partial f}{\partial \sigma }|}_{\sigma =\sigma_{1}}. \end{array}$$

Then the stress after adjustment can be determined using

(7) $$\begin{array}{c} \sigma =\sigma_{ij}=\left(1-n\right)\sigma_{ij}^{1}+p\delta_{ij}, \end{array}$$

where

(8) n=wμJ2,  p=−mw+3nI1,m=α(3λ+2μ),  w=f3αn+μ,

where *J*_2_, *I*_1_, and *f* can all be determined by *σ* and *λ* and *μ* are Lame constants, which can be expressed using

(9) $$\begin{array}{c} \lambda =\frac{E\nu }{\left(1+\nu \right)\left(1-2\nu \right)},\;\;\mu =\frac{E}{2\left(1+\nu \right)}. \end{array}$$

*E* and *ν* are Young's modulus and Poisson's ratio, respectively. Stress increment of each incremental step or iteration can be written in

(10) $$\begin{array}{c} \Delta \sigma^{p}=\sigma_{1}-\sigma =n\sigma_{ij}^{1}-p\delta_{ij}. \end{array}$$

#### 3.2.2. Numerical Model and Analysis Cases

Figure 5 depicts the numerical model for the Xiluodu arch dam, which consists of the whole dam structural and the foundations including faults and main weak zones such as the interstrata bedding planes C9, C8, C7, C3, C2, and C1 and the intrastrata rupture belts Lc6 and Lc5. The 3D finite element mesh includes a vast area of abutments and its size is 1500 m × 1000 m × 660 m (length × width × height). The total number of elements is 104785 with 6096 elements for dam body, 1890 elements for the surface outlets, 420 elements for the side outlets, and 1890 elements for the bottom outlets, where the dam toe block in the downstream side is marked using brown colour, as shown in Figure 5(a). The numerical method proposed in Section 3.2.1 was employed to perform the finite element analysis and study the outlet cracking and failure behaviour.

The 3D finite element nonlinear analysis was executed for the Xiluodu arch dam in the following analysis cases.

1. Case A: the whole dam under usual loads (i.e., the hydrostatic pressure, silt pressure, and gravity) and overloads (i.e., the hydrostatic pressure, silt pressure, gravity, and two to six times upstream water pressure).
2. Case B: dam without outlets, under usual loads and overloads.

It should be noted that in the analysis case A, the existence of sluice is not considered and there is no hydrostatic pressure in the area of the outlets.  Table 3 summarized physical-mechanical parameters adopted by the numerical simulation. The self-weights of the dam and abutments, the normal water loads at the upstream and downstream sides of the dam, and the temperature load are the main loads taken into account during these analysis cases. The elevation height of the water in the upstream side, the silt, and the water in the downstream side is 600 m, 490 m, and 378 m, respectively.

### 3.3. Effects of Outlets on Dam Deformation

For the analysis cases A and B, the displacement distribution in the upstream sides of the dam under normal loads is illustrated in Figures 6(a) and 6(b), respectively. Moreover, the displacements at the critical locations of the dam for the both analysis cases are summarized in Table 4.  Figure 7 depicts the variation of the displacement at the dam crown for both analysis cases under various overload conditions.

It is known from the numerical results that (1) under the normal loading conditions, the maximum displacements of the dam crown decrease slightly when the outlets are taken into account. The maximum displacement decrease is about 1.6 mm, as shown in Table 4. Thus, the outlets in the high arch dam may help shift the arch thrust force to both abutments and increase the transverse deformation. (2) The symmetry of the displacement distributions is good for both analysis cases A and B, which indicates that the dam abutments have good overall stiffness. For the analysis case A, the maximum displacements of the crown (Figure 7(a)), left arch abutment, and right arch abutment along the river flow direction were 106.9 mm at EL 520 m of the downstream surface, 27.4 mm at EL 400 m of the downstream surface, and 29.57 mm at EL 400 m of the downstream surface, respectively. For the analysis case B, the maximum displacements of the crown (Figure 7(b)), left arch abutment, and right arch abutment along the river flow direction were 108.5 mm at EL 520 m of the downstream surface, 28.7 mm at EL 400 m of the downstream surface, and 30.2 mm at EL 400 m of the downstream surface, respectively. (3) In the analysis case B, the dam body shoulders greater pressures from the water and silt at the upstream side. The carrying capacity of the arch fails to increase relatively while that of beam becomes heavier. These factors contribute to the increase of the displacement of the crown compared with the analysis case A.

### 3.4. Effect of Outlets on Dam Stress Distribution

In the design of the dam outlets, it is vitally important to investigate clearly the stress distributions in both dam and outlet, especially in the tensile zone at the roof, floor, and side walls of the outlets. Correspondingly, the distributions of the major and minor principal stresses at the upstream and downstream surface of the dam are depicted in Figure 8 for the analysis cases. The maximum tensile and compressive stresses of the dam and outlets are summarized in Table 5 for the analysis cases A and B under normal loading conditions, which include the hydrostatic pressure, silt pressure, and gravity.

It can be seen from Figure 8 and Table 5 that (1) the values of characteristic stresses such as the maximum tensile stress and the maximum compressive stress from both analysis cases are nearly the same, which indicates that though the dam body in the analysis case B carries more pressure from the water and silt in the upstream side because of ignoring the existence of the outlets, this small proportion of incremental pressure does not make much difference. The maximum compressive stress at the downstream surface in the analysis case B is 17.1 MPa, which is 0.2 MPa bigger than that from the analysis case A. (2) As for the maximum tensile stress at the upstream surface of the outlets, it is found that the upstream surface of the outlets in the analysis case B is slightly compressive while that in the analysis case A suffers from some high tensile stress. The surface outlet in the analysis case A is most likely to crack since the tensile stress there reaches 1.8 MPa. (3) Under the normal loading condition, the optimal distribution of the outlets in the arch dam will contribute to the release of the tensile stress concentrated in the local zone of the upstream surface and decrease the cracking risk of the integral dam body during the operation period. At the same time, stronger concrete and appropriate reinforcement measures should be used in the area near the outlets. (4) The results from the stress analysis and the displacement analysis are consistent with each other. If the outlets are filled, the elastic modulus of the filled outlets is increased, or the elastic modulus of the dam body is increased, the load carrying capacity of the arch dam improves significantly, especially in the part where the middle and bottom outlets are located. However, the tensile and compressive stresses at the left and right ends of the arch dam become larger.

Figures 9 and 10 show the distribution of the major and minor principal stresses in various parts of the bottom outlets from the analysis case A. It can be seen that the side walls and the roof are mainly under compression during the operation period but the tension stresses concentrate in the area close to the upstream side of the roof. Compressive stresses dominate the floor of the bottom outlets.

### 3.5. Effect of Outlets on the Integral Stability of the Arch Dam

The yield process of the arch dam at ultimate limit states is predicted by applying overloads on the dam in the analysis cases A and B. Figures 11(a) and 11(b) depict the yield zones in the horizontal sections of the middle outlets when the applied load is 6 times normal water load in the analysis cases A and B, respectively, while the yield zones in the upstream and downstream surfaces are shown in Figure 12. It can be seen that the yield zones are located in the downstream surface of the dam and showed a “butterfly” symmetrical distribution (Figures 12(a) and 12(c)). Compared with the analysis case A, the analysis case B generates a more widely distributed yield zone and a higher yield value. Therefore, filling the outlets decreases the carrying capacity of the dam body.

For the analysis case A under normal loads, there is no yield zone occurring in either the upstream or downstream surfaces. The factor of safety at various locations of the upstream surface is between 2.0 and 5.0. It is discovered from the sequentially overloading process that when the applied load is two times the normal load, a small yield zone appears in the heel of the upstream surface. As for the downstream surface, the yield zone spreads quickly under overload conditions and a large area becomes yield when the applied load reaches 4 times the normal water load.

For the analysis case B under normal loads, there is again no yield zone in either the upstream or downstream surfaces. The factor of safety at various locations of the upstream surface is between 2.0 and 5.0, too. The sequential overloading process in the analysis case B shows that when the applied load is two times the normal load, a small yield zone appears in the dam heel while some big yield zone appears in the downstream surface. As the times of the applied overload increase, the yield zone in the downstream surface spreads quickly. When the applied load reaches 3 or 4 times the normal water load, large yield zone appears in the downstream surface and the arch dam enters into nonlinear deformation stage, which indicates the beginning of the dam destruction.

It can be seen from the analysis cases A and B that the outlets are integral and help dam shoulder some load although they relatively weaken the carrying capacity of the arch dam. The initial cracking overload coefficient K1 is 2 and the ultimate overload coefficient is 6.5~7. It is obvious from above analyses that, under the overloading conditions, the cracks initiate around the outlets, propagate along the horizontal direction, and then coalesce in the area between the adjacent outlets. The yield zone generated in the dam under overloading conditions looks like a butterfly.

## 4. Outlet Cracking Mechanism and Risk Control

### 4.1. Outlet Cracking Mechanism

Based on the case studies on the outlet cracking in the Goupitan arch dam and the Xiaowan arch dam presented in Section 2 and the numerical simulation on effect of outlets on overall stability of the Xiluodu arch dam introduced in Section 3, it can be seen that the following factors contribute to dam outlet cracking: dam structural design, construction materials, thermal control, maintenance processes, and the impounding scheme. Potential reasons of the outlet cracking can be summarized as follows.

(*1) Concrete Materials*. Outlets are always part of the hydraulic structures, which are usually built with stronger concrete so as to improve the abrasion-resistant ability. However, the stronger the concrete is, the more the cement is used, which may generate the larger amount of hydration heat and the higher temperature. All these factors set higher requirements for the construction environment, temperature control, and maintenance measures. Cracking may easily occur once the temperature in the construction environment changes sharply, for example, the drop of the temperature in the late maintenance phase. In addition, if the concrete used in the bottom outlets differs sharply from that used in the surrounding dam body, that is, the shrinkage coefficients of the two kinds of concretes vary greatly, the risk of cracking still increase even if several different kinds of concretes are used in the transition zone.

(*2) Temperature Control and Maintenance*. Temperature control and maintenance of the concretes used to construct the outlets are relatively more complex than the other factors. In addition to conventional measures of the temperature control, the surface of the outlets has to be closed so as to prevent them from impact of low temperatures caused by cavern drafts flowing and water is kept to flow on the surfaces of the dam body concrete. If the measures of the temperature control and maintenance are not carried out properly, thermal cracking may easily occur in the outlet concrete due to temperature gradients.

(*3) Impounding Scheme*. During the construction phase, the water pressure in the reservoir influences the stress distribution in the dam. If the reservoir water is stored too early or too much, large tensile stresses may be induced in the upstream surface, heel, and shoulder of the dam. If the water storage is delayed, cracking may easily be caused by the tensile stress in the upstream face of the crown cantilever, which has large upstream-tend displacement. Thus, reasonable storage scheme should be figured out. During the construction phase of the arch dam, the concrete structure above a certain elevation belongs to a beam structure instead of an arch beam structure since the joints grouting of the arch dam only happens after the temperature of the dam body drops to a specified temperature.

(*4) Design Scheme*. Since the outlets may experience obvious deformation and are prone to tensile stress, reinforcement design is often required. Because of the complex structure and the big size difference from the dam body to the outlets and the effects on the outlets caused by the dam weight, water pressure, temperature gradient, concrete creep behaviour, and so on, the accurate analysis of stresses on the outlets becomes very difficult. So, the design scheme itself alone could not reduce the cracking risk effectively.

(*5) Concrete Fracture Characteristics*. According to the experiment on fracture properties of full graded concrete used in Xiluodu high arch dam, the initial fracture toughness of the concrete with one month age is 0.3 MPam^1/2^ in average, the unstable fracture toughness is 1.225 MPam^1/2^ in average, and the cracking toughness is 448.257 N/m in average. The corresponding values of the concrete with three months of age are 0.655 MPam^1/2^, 1.387 MPam^1/2^, and 470.600 N/m, respectively. Because of the low cracking-resistance ability of the early concrete and the complex conditions in the construction sites, the concrete dam is prone to generate initial microscopic cracks, especially around stress concentrated area like the outlets. The analysis conducted above shows that the cracks around the outlets have little impact on the dam integral stress and displacement but these cracks may propagate to coalesce with the interior temperature cracks and traverse joints and become the main source of the water leakage. The irregular cracks on the wall of the outlet corridors may propagate under the high pore water pressure in the cracks. Once these cracks propagate into deep depth or through the foundation and their direction is parallel to the axis of the dam, the consequences may be unbearable. In this case, these cracks may harm the dam structural integrity, change the stress condition of the concrete structure, and damage some local dam structures. Moreover, the durability of the concrete may be weakened. Thus, the effects of the superposition of the thermal and structural stresses on the integral stability of the dam allow no ignorance.

(*6) Outlet Cracking Risk*. Based on the case studies on outlet cracking in the Goupitan and Xiaowan arch dams, the diversion outlet is prone to local stress concentration and crack initiation due to hydration heat associated with the exothermic chemical reactions in the fresh concrete. Thus, the local reinforcement design is needed for the diversion outlet, which will be discussed in the next section. During the operation period, the stress and deformation distribution around the outlet generally satisfy the operation requirement of the dam under normal loading conditions. The outlets mainly affect the overall stability of the dam under overload conditions, especially when the yield zones occur around the outlets under the overloading conditions.

### 4.2. Cracking Risk Control and Reinforcement

#### 4.2.1. Experiences from Processing the Outlet Cracking in the Goupitan Arch Dam

Based on the case studies and the numerical modelling, crack reinforcement measures are proposed to repair the outlet cracks in the Goupitan arch dam.

As introduced in Section 2.1, the cracks inspected in the Goupitan arch dam can be classified into four types as shown in Table 1. Depending on the types of the cracks, the cracking treatment measures include surface processing, shallow processing, and deep processing.

(1)* The surface processing* is involved in brushing waterproof materials on the cracks, which is suitable for the cracks that have not gouged at the time of the inspection. (2)* The shallow processing* is involved in sealing and backfilling the cracks with preshrunk mortar and filling the grooved part of cracks with imperial materials during the inspection. (3)* The deep processing* is used to repair deep cracks, that is, to use chemical grouting method to reinforce the crack. After the chemical grouting, a site investigation should be done to inspect the surfaces of the repaired cracks. Moreover, the grouting quality should be examined by core-sample drilling and hydraulic pressure tests in 28 days after the chemical grouting. The samples from the core drilling should be tested to obtain the compressive resistant capacity and splitting resistant capacity besides the visual inspections. The testing results of the Goupitan arch dam show that the compressive resistant capacity of the sample taken from the core drilling after the chemical grouting is more than 40 MPa and the splitting resistant capacity is more than 2.0 MPa. The hydraulic pressure tests are conducted using the holes from the core drilling or those drilled alone and the pressure of the injected water during the inspection is 0.2 MPa. It is found that the results from the hydraulic pressure tests satisfy the judgment standard, which allows no more than 0.1 Lu permeation rate. In addition, the deep sonic wave tests are also conducted after the grouting is completed, whose results are compared with those from the visual inspection and the tests mentioned above so as to have a further examination of the grouting quality.

#### 4.2.2. Experiences from Processing the Outlet Cracking in the Xiaowan Arch Dam

The outlet cracking in the Xiaowan arch dam has been reinforced in two times. The reinforcement measure in the first time is intended to repair the cracks in the middle diversion outlets which happened before August 2008. At that time, the cracks due to the temperature gradients have not been observed and the cracks in the middle diversion outlets have not coalesced with those due to the temperature gradients yet. The reinforcement measures include grooving the cracks and spraying impervious materials on the surfaces of the cracks.

The reinforcements in the second time happened in May 2009, when several cracks in the middle diversion outlets had been found to coalesce with the cracks due to the temperature gradients. The main reinforcement measures include chemical grouting and grooving and spraying impervious materials on the surface of the cracks, which can be detailed as follows: (1) grooving and backfilling with preshrunk mortar immediately. (2) For the water leakage cracks, a 4 mm thick polyurea coating is sprayed in the scope of 2 meters around the cracks. For the area with dense cracks, the 2 m scope is determined from the crack located in the edge of the area. (3) Chemical grouting is applied in the cracks, which coalesce with the thermal cracks due to the temperature gradients inside the dam.

#### 4.2.3. Principles for Outlet Cracking Risk Control and Reinforcement in the Super-High Arch Dam

In this section, a reinforcement principle is proposed to control the outlet cracking risk based on the reinforcement experiences of the outlet cracking in the Goupitan and Xiaowan arch dams in Sections 2, 4.2.1, and 4.2.2 and the numerical studies on the effect of the outlets on the integral stability of the Xiluodu arch dam in Section 3.

(*1) Selection of Appropriate Concrete Materials*. The dam outlets are a hydraulic structure for water diversion, which should be designed using the concretes with appropriate strengths according to their flow rate. The concrete with high strengths should not be used blindly. If the abrasion-resistant capacity of the concrete is only to be improved, the fibre-reinforced concrete may be used, which may reduce the use of the cement then lower down the hydration heat and alleviate the pressure from the temperature control. If the outlet must be constructed using the high strength concrete, whose expansion coefficient is much different from that of the concrete used to construct the dam body, a transition area must be constructed between the outlets and the dam body using various types of concretes and the expansion coefficients of the adjacent concretes should not differ significantly.

(*2) Strengthening Temperature Control during Construction Period*. The routine temperature control measures should make sure that the temperature of the concrete in each procedure satisfies the requirement including the concrete mixing and pouring temperatures, the highest temperature inside the concrete, and the temperature difference between the inner and external surfaces of the concrete. The concrete may be poured under low ambient temperatures such as nighttime. Special temperature control measures may be adopted for the bottom diversion outlets: (1) the concrete started to pour from the outlets. The surfaces of the outlets may be closed using curtain-style closed doors to prevent the surface of the concrete from the wind blowing through them, which may reduce the temperature of the concrete, result in too high temperature gradient, and induce thermal cracking. (2) When the mould at the sidewalls of the outlet is dismantled, thermal insulation quilt with 2 cm thickness should be installed to maintain the temperatures there. (3) Canvas insulation frame is installed at the upstream and downstream sides of the outlets to maintain the temperatures when the outlets are formed. (4) When the construction of the floor of the bottom diversion outlet is finished, water flow is used to maintain the temperatures there, which may be replaced with watering in 1 or 2 days after the highest temperature of the poured concrete appears.

(*3) Reasonable Impounding Scheme*. The impounding scheme should make sure that the reservoir is impounded with water as early as possible when the stress state and the point factor of safety of the dam body and the outlets satisfy the design requirements. In this case, the height of the cofferdam can be reduced as low as possible and the electricity can be generated as early as possible.

(*4) Optimizing Outlet Design*. The outlets should be designed to reduce the size of the tensile stress, which may appear near the outlets, and the area of the outlet, which may be under tension, in order to reduce the reinforcement as far as possible. The potential engineering measures may include changing the shape of the outlets, grouting the transverse joints, filling and pressuring the transverse joints, and preloading and grouting aggregates. Moreover, physical model testing and numerical modelling may be conducted to study the stress and strain characteristics of the outlets, the progressive development of the outlet crack initiation, propagation and coalescence, and the nonlinear reinforcement method for the outlets.

(*5) Outlet Cracking Classification and Reinforcement*. Based on the case studies and numerical simulations conducted above and the arch dam design code, the outlet cracking can be classified and reinforced according to the following engineering procedure: cracking investigation → causes of cracking and cracking category analysis → hazard evaluation and classification → patching treatment → inspection and acceptance.

## 5. Conclusions

This paper first conducts two case studies on the outlet cracking in the Goupitan and Xiaowan arch dams by focusing on the current statuses, reasons, and potential consequences of the dam outlet cracking. Then, effect of outlets on the integral stability of the Xiluodu super-high arch dam under normal loading and overloading conditions is studied using 3D nonlinear finite element method. After that, the outlet cracking mechanism and risk control are discussed on the basis of the two case studies and numerical modelling. Finally, a reinforcement principal is proposed to control the dam outlet cracking risk. The following conclusions can be drawn.

1. Special attention should be paid to the effects of the outlets on the working conditions of the super-high arch dam. It is found that the outlets decrease the upstream pressure of water and sand/silt and the dam stress, longitudinal displacement, and transverse displacement. The maximum reduction ratio can be 35%. Thus the outlets may harm the structural continuity of the arch dam, weaken the carrying capacity, and decrease the load pressing on the dam surface.
2. Under normal loading conditions, the optimal distribution of the outlets will contribute to the tensile stress release in the local zone of the stream surface and decrease the cracking risk under operation period. Under overloading conditions, cracks initiate around the outlet then propagate along horizontal direction, and finally coalesce with the adjacent outlet cracks. The yield zone of the dam has a shape of a butterfly. The integral bearing capacity of the dam may increase about 20% if the elastic modulus of the concrete used for the outlet increases.
3. The outlet cracking is caused by many factors including the concrete materials, temperature control and maintenance, impounding scheme, and dam design scheme.
4. A reinforcement principle is proposed to control the outlet cracking risk through selecting the appropriate concrete materials, strengthening the temperature control during construction period, designing reasonable impounding scheme, optimizing the outlet design, and classifying the outlet cracking for various reinforcement measures.

## Figures and Tables

**Figure 1:** Distribution of the outlets of the Goupitan arch dam.

**Figure 2:** Schematic sketch and photo of outlet cracking in the number 1 reservoir empting bottom outlet of the Goupitan arch dam.

**Figure 3:** Schematic sketch of outlet cracking in the number 2 reservoir empting bottom outlet of the Goupitan arch dam.

**Figure 4:** Cracking near the middle diversion outlets of the Xiaowan arch dam.

**Figure 5:** 3D mesh model of dam and outlets.

**Figure 6:** Displacement contour along river direction under different analysis cases (normal loads).

**Figure 7:** Crown displacement along river direction under various analysis cases (overloading condition).

**Figure 8:** The principal stress distribution (analysis case A; Unit: pa; “−” denotes compression stress, and “+” denotes tension stress).

**Figure 9:** The first/third principle stress distribution of bottom outlets under analysis case A.

**Figure 10:** The first/third principle stress distribution of bottom outlets under analysis case A.

**Figure 11:** Plane section of yield zone in middle outlets under various analysis cases (6 times overloading).

**Figure 12:** Yield zone in dam under various analysis cases (6 times overloading).

**Table 1:** Cracking characteristics and reinforcement measures of the numbers 1 and 2 reservoir emptying outlets in the Goupitan arch dam.

Outlets	Series number	Cracking depth (m)		Cracking description	Reinforcement measures
		Max	Min		
Number 1 reservoir emptying bottom outlet	Crack series number 1	0.3	0.3	Deck of the number 13 dam monolith at EL 491 m	Groove in cracking surface Fill in cracks using preshrinkage mortar Embed grouting pipe system Drill stress release hole Install double-layer crack-limiting steel bar
	Crack series number 2			From EL 494 m to EL 488 m along the number 13 dam monolith	
	Crack series number 3	1.1	0.7	Deck of the number 14 dam monolith at EL 497 m	
Number 2 reservoir emptying bottom outlet	Crack series number 1	1.5	0.3	Deck of the number 14 dam monolith at EL 497 m	
	Crack series number 2			From EL 494 m to EL 488 along the number 13 dam monolith	
	Crack series number 3	1.7	0.3	Deck of the number 15 dam monolith at EL 490 m	
				Deck of the number 15 dam monolith at EL 494 m	

**Table 2:** Cracking characteristics and reinforcement measures of the middle outlets in the Xiaowan arch dam.

Location	Crack number	Depth of cracks (m)		Cracking description	Reinforcement measures
		Max	Min		
Number 21 dam monolith (number 1 diversion outlet)	21LF-1	1.2	0.3	Cracks are distributed at ring shape in the dam monolith from EL 1012 m~1110 m. There are 19 cracks with length less than 3 m in the left side wall of the number 1 middle diversion outlet at the downstream side and 1 microcrack with length smaller than 2.3 m in the right sidewall	Crackings around the diversion middle outlets have been inspected before August 2008. At that time, these cracks did not coalesce with the thermal cracks caused due to temperature gradients, which were not completely identified. The reinforcement measures were cracking filing and surface permeable-resistant coating It was noted that cracks around the diversion middle outlets have coalesced with the thermal cracks due to temperature gradients till May 2009. The main reinforcement measures include chemical grouting, crack filling, and surface permeable-resistant coating, which are detailed as follows (1) Cracks are grooved and filled (2) Surface permeable-resistant coating: the surface of the dam monoliths is coated using impermeable polyurea with a thickness of 4 mm in 2 m around the cracks. For the area with the dense fine cracks, the 2 m is counted from the crack located in the boundary of the area (3) Chemical grouting is applied in the cracks which coalesce with the thermal cracks due to temperature gradients
	21LF-2	1.7	0.3	In April 2009, a crack with a length of 29 m along the flow direction was found in the floor of the number 1 middle diversion outlet at the upstream side, which perpendicularly intersected with thermal cracks due to temperature gradients. No cracks were found in the roof and side walls	
Number 22 dam monolith (number diversion outlet)	22LF-1	1.1	0.3	Cracks are distributed in the number 22 dam monolith between ELs 1068 m and 1098 m but above the floor of the number 2 middle diversion outlet whose EL is 1065 m	
	22LF-2 22LF-3	1	0.2	Cracks coalesce with surface cracks in the number 2 middle diversion outlet. The cracks 22LF-2 are distributed in the number 22 dam monolith at ELs between 1013 m~1050 m. The cracks 22LF-3 are distributed above 5 m~7 m below the cracks 22LF-2 Large number of irregular microcracks were observed to distribute in ring shape in the floor, side walls, and roof of the number 2 middle diversion outlet between the thermal cracks 22LF-2 and 22LF-3 in the second-round inspection of the outlets in February 2009.	
	22LF-4	1	0.3	The cracks lie in the downstream side of the number 22 dam monolith between ELs 972 m~1012 m, which are expected to intersect with the surface of the dam monolith	
Number 23 dam monolith (number 3 diversion outlet)	23LF-1	1.7	0.5	The cracks are distributed in the number 23 dam monolith between ELs 1001 m~1108 m and extend through the number 3 middle diversion outlet	
	23LF-2	1.75	0.5	The cracks lie in the number 23 dam monolith between ELs 977 m~1025 m, which extend till 1021 m but have not reached the floor of the number 3 middle diversion outlet.	

**Table 3:** Physical-mechanical parameters of the rock masses and dam materials.

Materials	Bulk density (t/m^3^)	Deformation modulus (GPa)	Poisson's ratio	Shear strength	
				*C*′ (MPa)	*F*′
Dam concrete	2.40	24	0.167	5.0	1.70
Concrete of bottom outlets	2.40	32	0.167	5.0	1.70
Rock of class II	2.85	16.5	0.20	2.5	1.35
Rock of class III1	2.85	11.5	0.25	2.20	1.22
Rock of class III2	2.75	5.5	0.28	1.4	1.2

**Table 4:** Dam displacement at the downstream side along the river direction under various analysis cases (unit: mm).

Case	Level position (m)	610	590	560	520	480	440	400	360	332
Case A	Left arch abutment	5.3	7.8	15.2	18.2	23.8	23.7	27.4	27.2	23.7
	Arch crown	94.8	99.8	103.9	106.9	100.5	89.3	72.2	48.8	25.3
	Right arch abutment	3.5	5.1	10.4	15.6	20.4	25.5	29.5	25.4	21.2

Case B	Left arch abutment	5.7	7.9	15.3	18.7	24.3	23.9	28.7	28.2	24.3
	Arch crown	95.3	100.4	104.7	108.5	102.3	90.9	73.7	50.2	26.7
	Right arch abutment	3.7	6.4	11.7	16.7	21.4	26.9	30.2	26.3	21.4

**Table 5:** Characteristic stresses at various key locations from both the analysis cases A and B (Unit: MPa).

Location	Content	Case A	Case B
Up stream surface	Maximal tensile stress of dam heel	0.67	0.85
	Maximal tensile stress near left arch abutment	0.61	0.82
	Maximal tensile stress near right arch abutment	0.1	0.1

Down stream surface	Maximal compression stress of dam toe	15.7	16.8
	Maximal compression stress near left arch abutment	16.9	17.1
	Maximal compression stress near right arch abutment	16.3	16.7

Upstream of bottom outlet	Maximal tensile stress of side wall	−1	—
	Maximal tensile stress of roof	0	—
	Maximal tensile stress of floor	−0.1	—

Downstream of bottom outlet	Maximal tensile stress of side wall	0.7	—
	Maximal tensile stress of roof	0	—
	Maximal tensile stress of floor	0	—

Surface outlets	Maximum tensile stress in upstream surface	1.8	—
	Maximum tensile stress in downstream surface	1.9	—

Middle outlets	Maximum tensile stress in upstream surface	1.5	—
	Maximum tensile stress in downstream surface	1.7	—
